The article "The Regulation of miR-206 on BDNF: A Motor Function Restoration Mechanism Research on Cerebral Ischemia Rats by Meridian Massage" was published in 2022. Journal: Evid Based Complement Alternat Med.

# The Regulation of miR-206 on BDNF: A Motor Function Restoration Mechanism Research on Cerebral Ischemia Rats by Meridian Massage

**DOI:** 10.1155/2022/8172849

**Published:** 2022-08-27

**Authors:** Guofeng Shi, Ping Zeng, Qing Zhao, Jinju Zhao, Yunhui Xie, Danguo Wen, Lu Yan, Hao Gu, Shuai Ma, Xiongwei Cai

**Affiliations:** ^1^Guizhou University of Traditional Chinese Medicine, Guiyang 550000, Guizhou, China; ^2^Southwest Hospital, Army Medical University, Chongqing, China

## Abstract

As a frequent disease affecting the nervous system, cerebral infarction has emerged as a major cause of disability and elicits disorders in motor, sensation, and cognition as sequelae. No clear mechanism has been known in meridian massage despite it having been proved to be an effective therapeutic option. The study was carried out to explore the treatment of meridian massage on cerebral ischemia in rats and its effects on motor function restoration and nerve cell's ultrastructure in the ischemic territory. The alleviated nerve damages and recovered injured brain tissues were found in the cerebral infarction model of SD rats after meridian massage. Expressions of miR-206 and the brain-derived neurotrophic factor (BDNF) in the gastrocnemius muscle were all well observed. The effects of miR-206 on BDNF were testified by overexpressed and interfered miR-206 in the C2C12 myoblast. Moreover, at the molecular level, meridian massage downregulated miR-206 expression at an elevated level of BDNF. Consequently, meridian massage exerts a vital role in promoting cerebral ischemia restoration, which is expected to provide an addition to the application of traditional Chinese medicine (TCM) in the reconstruction and treatment of cerebral ischemia.

## 1. Introduction

Cerebral infarction, a common disease affecting the nervous system, has evolved into the top three lethal diseases causing mortality [1]. Despite the risk of stroke dropping by 25% till 2010 as medical technologies and methods advanced, the rate of disability remains on the rise even over 80%, struck by sequelae, namely, motor, sensory, and cognitive disorders, which become a heavy burden carried upon the shoulders of patients, their families, and society [2, 3]. Early formal training on functional rehabilitation has been proved effective in the restoration and improvement of the motor function after episodes of cerebral infarction living a better quality of life for patients. Of all the therapies, meridian massage manifests a satisfactory efficacy in clinical application, while little has been revealed on its working mechanisms. In light of the meridian-collateral theory in traditional Chinese medicine (TCM), meridian massage in combination with the naprapathy principle treats diseases employing conducting meridians and relieving muscle spasms, thus stimulating muscles to produce a passive movement and regulating Qi and blood in viscera [4–6]. Our team has made clinical achievements with the application of meridian massage which ameliorates the motor function of patients suffering from cerebral infarction. An interference of rehabilitation training alters the expression patterns of angiopoietin, Nogo-A, and brain-derived neurotrophic factor (BDNF) and facilitates axonal bud synaptic reconstruction for the recovery of functions in the brain and loops [7]. In addition, the therapy of rehabilitation training promotes the proliferation of glial cells, vascular endothelial cells, and macrophages around necroses and accelerates necrosis reconstructions, thereby advancing compensatory effects of normal tissues and facilitating the recovery of the motor function [8, 9]. Clinically, meridian massage in an early stage of rehabilitation training produces an efficient outcome in improving the cerebral blood flow of acute cerebral infarction patients through strengthening motor function recovery and enhancing the paralyzed limb functions. In addition, early training on functional rehabilitation contributes to a prominent result. Most studies on the mechanism of meridian massage on motor function reconstruction after cerebral infarction give priority to cerebral microangiogenesis, neurotrophic factors, and various brain-protective proteins, while the mechanism of meridian massage in promoting skeletal muscle recovery remains to be explored.

Neurotrophic factors present as proteins that maintain functions, support the survival of the neurons, and promote cell growth as well as differentiation [10]. Myogenic neurotrophic factors are possibly uptaken by the motor nerve axon terminal and retrograde transported to neuronal somas, which affects the survival and differentiation of motor neurons and exerts vital importance in the development and function maintenance of neuromuscular junction (NMJ) [11, 12]. The neurotrophic factors related to motor neurons include neurotrophins and BDNF, among which BDNF functions as one of the crucial members in the neurotrophic family and produces an essential role in neuron survival, growth, differentiation, neurotransmitter release, and synaptic plasticity [13–15].

The miRNA regulation of genes is speculated to contribute to the performance of highly complex functions for vertebrate muscles, and the specific expression of miR-206 has been reported in skeletal vertebrate muscles and high expression in slow muscles [16]. Accordingly, it may regulate gene expression as muscle satellite cells develop and muscle fiber types converse in adult animals. Most miRNAs inhibit the translation of target genes in the cytoplasm, while the expression of miR-206 is noticed in the cytoplasm and nucleus of myoblasts. The unique expression pattern indicates a significant role of miR-206 in skeletal muscle pathophysiology, which requires further study in pursuit of the significance of miR-206 and other molecules during the course.

More investigations suggest that miR-206 regulates the expression of the BDNF which means the inhibition of miR-206 increases the level of BDNF [16]. By mediating multiple functions of synaptic plasticity, the BDNF plays a role in improving cognitive function, neurogenesis, as well as neuronal differentiation. Studies in Alzheimer's disease (AD) rats have demonstrated that increased levels of brain-derived neurotrophic factors and the administration of AM206 and miR-206 blocker, both may enhance the expression of hippocampal synaptophysin and neurogenesis and cognitive function [17]. The expression of miR-206 indicates an upregulation in the frontal cortex during cerebral ischemia. In normal circumstances, the level of miR-206 is undetectable or too low to be detected in the brain, while it is highly expressed in neurological-related diseases, suggesting that miR-206 might participate in the pathogenesis of AD by inhibiting the BDNF expression, thereby affecting motor function [18–20]. So, the maintenance of miR-206 at an appropriate physiological level is proved to be of great significance. Exercise experiments have revealed that the miR-206 expression is high in a quiet state but the level is reduced through a chronic endurance exercise. After the training, the miR-206 expression falls back to the former level, implying that miR-206 may directly alter the physiological effects of human endurance sports, that is why miR-206 is known as a skeletal muscle function regulator. As mentioned in the previous study, meridian massage may act as an external force on muscle tissues, facilitating expressions of BDNF and inhibiting miR-206 in muscles, thereby improving the synaptic function of neuromuscular junctions and easing the dysfunction by recovering the impaired motor function. Based on the previous research, this study has been established to dig out the effects of meridian massage on the reconstruction of the motor function, the ultrastructure of nerve cells in the ischemic territory, and the expressions of both miR-206 and BDNF in gastrocnemius muscles. We also aim to investigate the mechanism of meridian massage on motor function reconstruction after cerebral infarction to treat the rat models of cerebral infarction utilizing meridian massage therapy.

## 2. Methods

### 2.1. Animals

A total of 72 male SD rats weighing 250∼280 g were provided by the Chongqing Enswil Biotechnology Co., Ltd., 12 h–12 h day and night alternated. The animals were supplied with food and water at will at a temperature of 23–25°C, and the experiment was performed after adaptive feeding for one week. The experiment was approved by the ethics committee of Guizhou University of traditional Chinese medicine.

### 2.2. Animal Modeling and Sampling

The SD rats were anesthetized with 1% pentobarbital sodium (50 mg/kg) and fixed on the operation board with a medical tape in a supine position. The skin of the neck of the rats was shaved and disinfected with an alcohol swab. A 2∼3 cm cut was made in the skin in the middle of the neck, and the submandibular gland and right muscle were bluntly separated exposing the common carotid artery, which was carefully separated, and so did the vagus nerve. Internal and external carotid arteries were dissected with care, and the external carotid artery was ligatured. With the internal carotid artery being temporarily clamped by an arterial clamp, the distal end of the common carotid artery was ligatured. The 4–0 surgical suture was utilized for ligation with the common carotid artery elevated. A V-shaped cut was opened with a spring scissors and a special suture was inserted, slightly tightening the prepared suture to avoid blood reflux. No resistance caused by the insertion of the tethered wire was felt until the mark of the tethered wire reached the bifurcation of the common carotid artery and internal carotid artery if the wire entry was smooth. Then, a slight resistance could be felt at the tip of the tethered wire; then, we stopped plugging and ligated the prepared line. Muscles and skins were sutured layer by layer, disinfected with cotton balls containing alcohol, and the rats were put back into the cage. The rats were anesthetized 1.5 h after surgery the neck was disinfected and then cut with an open. Ophthalmic tweezers were employed to clamp the sites to be sutured. The suturing line was pulled out to the head and cut the excess before being sutured layer by layer and sterilized. As for the sham operation group, only the common carotid artery was dissected and sutured immediately. The rats were placed back in their cages after the operation supplied with sufficient feed and water.

The rats were randomly divided into the model group, meridian massage group, and sham operation group, with 24 in each group. Twenty-four hours after the successful establishment of the middle cerebral artery occlusion (MCAO) rat model, the rats from the model group and the sham operation group were kept in ordinary cages, no rehabilitation training was given but food, water, and movement were at their will. Conversely, the model group + meridian massage group were given meridian massage for 21 days. According to the positioning standards of Experimental Acupuncture Science and Chinese Veterinary Acupuncture Science, the rats were massaged at the Biguan (ST31), Taichong (LV3), Fenglung (ST40), and Zusanli (ST36) acupoints, with the emphasis on the gastrocnemius muscle and the back of the thigh [21]. The rats' limbs were slightly hot and able to bear for 10 min, twice a day, for 21 consecutive days. The SD rats in each group were anesthetized with 7% chloral hydrate (0.5 mL/100 g) after 3, 7, 14, and 21 days, respectively, before samples were collected as below after successful anesthesia.

The whole blood: The abdominal cavity of the rats was opened and the abdominal aorta was located. One sample of whole blood was collected with an anticoagulation vacuum blood collection tube for the subsequent extraction of leukocytes. Another whole blood sample was collected with a non-anticoagulation blood collection tube and centrifugated. The supernatant was collected and stored at −80°C. The gastrocnemius muscle: Following the blood collection, the gastrocnemius muscle was dissected, washed with PBS, and then stored at −80°C for later use. The brain: The chest cavity was opened and the apex of the heart was connected to the injection needle of the infusion bag. The right atrial appendage was cut off to perform heart perfusion. PBS perfusion was initiated until the lungs turned white, then switched to 4% of paraformaldehyde and continued the perfusion. Dura mater and the whole brain were removed. The hippocampus and hemiplegic lateral frontal lobe were isolated and kept for 48 h which were scheduled for section staining. The electron microscopy sample was switched with 2.5% glutaraldehyde perfusion after the PBS perfusion and the rest surgery parts were identical.

### 2.3. HE Staining

All washed samples were fixed with 4% paraformaldehyde, and these tissues were immersed in 75% ethanol, 85% ethanol, 95% ethanol I, 95% ethanol II, 100% ethanol I, and 100% ethanol II in an orderly fashion, each for 2 hr. The dehydrated tissues were then soaked in 1/2 xylene, xylene I, and xylene II, in turn, each for 10 min. After transparent treatment, tissues were immersed in melted paraffin for 3 h to make paraffin sections. Tissues made from paraffin blocks were cut into slices at a thickness of 5 *μ*m with a microtome, laid flat on the fall-proof glass, and placed in a baking machine at 55°C to ensure the tissue pieces were tightly attached to the sliding glass. The paraffin sections were initially soaked in xylene I, xylene II, and 1/2 xylene for 10 min each for dewaxation and then in 100% ethanol I, 100% ethanol II, 95% ethanol I, 95% ethanol II, 85% ethanol, and 75% ethanol for 5 min each. All samples were washed twice with distilled water for 2 min each time for a total of 3 times. Staining was performed with hematoxylin for 10 min. After that, tap water was utilized to rinse the excessive staining solution for about 5 min and then washed with distilled water. Of 1% of hydrochloric acid, alcohol was used to decolorize excessive hematoxylin staining solution in the cytoplasm. Eosin staining lasted 30 s. Running water was lasted for 3 min to remove the excessive staining solution, and it was washed with distilled water again and dehydrated with 95% ethanol twice, 2 min each time. Then, xylene was utilized for hyalinization twice, 5 min each time. The neutral resin was used for blocking. Microscopic examination displayed that the nucleus turned blue and the cytoplasm was either red or pink.

### 2.4. Transmission Electron Microscopy Observation

The samples were prefixed with 3% glutaraldehyde, re-fixed with 1% osmium tetroxide, and then dehydrated with acetone at concentrations of 30%  ⟶  50%  ⟶  70%  ⟶  80%  ⟶  90%  ⟶  95%  ⟶  100% (three times at 100%) in an orderly fashion. Permeation was conducted with a dehydrating agent and epoxy resin (model Epon812) successively at ratios of 3 : 1, 1 : 1, and 1 : 3, respectively. Each step lasted 30∼60 min. The infiltrated sample blocks were placed in an appropriate mold filled with embedding solution and embedded into a solid matrix (embedded blocks) for heating and polymerization. This preparation was performed for later use. About 50 nm thickness ultrathin slices were prepared by using an ultrathin slicer, which was available in floating on the liquid surface in the groove, which was transferred to a copper mesh, stained with uranium acetate first, followed by lead citrate, at room temperature for 15∼20 min, and observed with a transmission electron microscope (JEM-1400PLUS).

### 2.5. RNA Extraction and RT-qPCR

The total RNA was extracted with the TRIzol reagent (Thermo Fisher Scientific). cDNA was synthesized through the TaqMan® MicroRNA Reverse Transcription kit (Thermo Fisher Scientific) in line with the manufacturer's instructions of use. qPCR assay was performed to quantify amounts of miRNA and mRNA with iQ™ SYBR® Green Supermix (Bio-Rad Laboratories) through the iCycler iQ™ qPCR detection system (Bio-Rad Laboratories). Relative levels of miR-206 and BDNF were calculated as the inverse log of ΔΔCt and normalized to the reference genes. Thermocycling was set at the following conditions: 95°C for 10 min; followed by 40 cycles of 95°C for 15 sec and 60°C for 1 min; annealing at 55°C for 30 sec; and elongation at 72°C for 3 min. GAPDH was regarded as an internal control for the analysis of BDNF mRNA expression and U6 was deemed as the internal control for the identification of miR-206 expression. Primers included U6–F, CCTGCTTCGGCAGCACATAT; U6-R, GAACGCTTCACGAATTTGCGT; GAPDH-F, GCAAGTTCAACGGCACAG; GAPDH-R, GCCAGTAGACTCCACGACATA; mir-206-F, GCGGAGTGGAATGTAAGGAA; mir-206-R, GTGGAGTCGGCAATTCAGTT; BDNF-F, GTCCACGGACAAGGCAACT; and BDNF-R, CAGCAGCTCTTCGATCACG.

### 2.6. ELISA

The ELISA kit was utilized to detect the expression level of BDNF (RD, DY248). Blank wells, standard wells, and sample wells were set for determination. 100 *μ*L of the sample diluent was added to the blank wells Another 100 *μ*L of standard or test samples was added to the remaining wells. The reaction processes were performed at 37°C for 120 min. The liquid was discarded and spun dry. A 100 *μ*L working solution of biotinylated antibody was added to each well, incubated at 37°C for 60 min, with the supernatant being discarded and spun dry. The plates were washed 3 times after being soaked for 1–2 min each time, 350 *μ*L/per well, spinning dry. 100 *μ*L of horseradish peroxidase-labeled avidin working solution was added to each well and incubated at 37°C for 60 min. After that, the supernatant was discarded, spun-dried. The plates were rinsed 5 times after being soaked for 1–2 min each time, 350 *μ*L/per well, spun-dried. 90 *μ*L of the substrate solution was added to each well in an orderly manner and incubated at 37°C in the dark for 5–10 min. 50 *μ*L of the stop solution was added to each well in sequence to terminate the reaction. Successive measurement of the optical density of each well was carried out with an enzyme-linked instrument (Thermo Fisher Scientific) at a wavelength of 450 nm. Procedures were performed within 15 min after the addition of the stop solution.

### 2.7. Western Blot

Tissue samples were lysed with a radioimmunoprecipitation assay buffer (Beyotime, China). Protein concentrations were examined by using the BCA Protein Assay kit (Pierce; Thermo Fisher Scientific). A number of protein extracts (30 *μ*g total protein/lane) were resolved with 10% SDS-PAGE, transferred onto PVDF membranes, and blocked with 5% dried skim milk at room temperature for 1h. The PVDF membranes were incubated with the BDNF primary antibody (cat. no. BM1307; 1 : 500; IGEE) and *β*-actin antibody (cat. no. BM026; 1 : 1,000; IGEE) at 4°C overnight with gentle agitation, and then treated with horseradish peroxidase-labeled goat anti-rabbit secondary antibody (1 : 1,000; cat. no. BM003; IGEE) at room temperature for 2 h. *β*-Actin was served as a loading control. The protein bands were visualized by using an enhanced chemiluminescence system (Beyotime, China).

### 2.8. C2C12 Myoblast Culture

C2C12 myoblasts were cultured in a DMEM high-glucose medium (Sigma, China) containing 10% fetal bovine serum (Hyclone, USA) and incubated in a incubator with 37°C, 5% CO_2_, at a constant temperature, and the medium was changed every other day. When the cells are confluent and reach about 80% of the growth density, a negative pressure is formed through the cell flexible substrate-loading device to generate a tensile strain on the culture membrane, so that the adherent and growing cells are subjected to tension.

### 2.9. Luciferase Reporter Assay

Wild-type (WT) or mutant (MUT) BDNF-3′UTR containing miR-206 binding sites were inserted into the psiCHECK2 vector (Promega, USA). The 293 T cells (1 x 10^5^ cells/well) were co-transfected with 0.1 mg of psiCHECK2-WT BDNF-3′-UTR or 0.1 mg psiCHECK2-MUT BDNF-3′-UTR and 10 nM of miR-206 mimics or 10 nM of miR-206 inhibitors in a way of Lipofectamine® 2000 reagent (Invitrogen, USA) as per the manufacturer's instructions of use. Cells were cultured at 37°C for 48 h, whose luciferase activities were analyzed by using a dual-luciferase kit (Promega, USA) in terms of the manufacturer's instructions of use. The activity of firefly luciferase was normalized to corresponding Renilla luciferase activity.

### 2.10. Statistical Analysis

Results were presented as the mean ± SEM. Significance analysis was established by the SPSS 13.0 software. Data were analyzed according to Student's *t*-test or one-way analysis of variance followed by Tukey's honest significant difference test. *P* < 0.05 was considered a statistically significant difference.

## 3. Results

### 3.1. Meridian Massage Restored the Neuronal Cell Morphology and Structure of Cerebral Infarction in Rats

The cerebral infarction model of SD rats was established (Figures 1(a) and 1(b)). Observations were made on the morphology of the cerebral cortex and hippocampus by HE staining. No obvious changes were visible over time at the injured parts in cerebral cortex models, while nerve cell edema was displayed severely affected with an increasing perinuclear space, and inflammatory cell infiltration was also revealed in some interstitium. The degeneration of nerve cell edema at injured parts was significantly relieved over time in the treatment group (repeated massage) compared with the model group. Results of HE staining in the hippocampus revealed that nerve cells of the hippocampus took on a scattering distribution in the model group. Blurred contours of nuclear shrinkage cells were presented and various edemas were observed in the interstitium (Figure 1(c)). The alignment of nerve cells in the treatment group (repeated massage) turned regular gradually and arranged tightly as time passed by in comparison with the model group.

### 3.2. Meridian Massage Restored the Damaged Nerve Cells and Reduced Apoptosis and Autophagy

Structures of nerve cells in rats were observed in the sham operation group, the cerebral infarction model group, and the meridian massage treatment group via transmission electron microscopy. In the brain tissue samples of the sham operation group, nuclei of nerve cells presented round, chromatin was evenly distributed, the nuclear membrane was clear and complete, and the cytoplasm was rich in complete and clear ribosomes, myelin sheaths, microfilaments, and mitochondria, among which the nerve myelin sheaths were relatively compact (Figure 2). The model group featured characteristics of apoptotic cells: blurred brain samples, some necrotic nerve cells with loose structures, rupture of cell membranes, massive mitochondria swelling in the cytoplasm, disappearing cristae forming into vacuoles, aggregation of nucleus chromatin, integral nuclear membranes but with shrinkage cell volumes, denatured myelin sheaths of myelin nerve fibers and obvious autophagy. Results of the treatment group presented round nuclei of the nerve cells, evenly distributed chromatin, clear and integral nuclear membranes, mitochondria in the cytoplasm, rough endoplasmic reticulum, and ribosomes. Swelling occurrence and autophagy and apoptosis were distinctly reduced in the treatment group compared with the model group. The abovementioned findings attested to the therapy of meridian massage that restored nerve cell damage and reduced apoptosis and autophagy.

### 3.3. Meridian Massage Reduced the miR-206 Expression and Enhanced the BDNF Expression after Cerebral Infarction

Subsequently, we determined expressions of miR-206 and BDNF in separate samples of gastrocnemius muscles and whole blood in rats by qPCR on days 3, 7, 14, and 21; results indicated that the expressions of miR-206 in whole blood and gastrocnemius muscles ranked the top in the model group (Figures 3(a) and 3(c)), the second was the treatment group and the lowest was the sham operation group. Such findings provided opposite data against the expression patterns of BDNF (Figures 3(b) and 3(d)).

The expression of BDNF in gastrocnemius muscles was testified by western blot (Figure 4(a)). From the results of the grayscale analysis, we know that the BDNF was highly expressed in the sham operation group, followed by the massage group, and the last one was the model group (Figure 4(c)). The expression of BDNF in gastrocnemius muscles was subjected to ELISA. BDNF expression results exhibited 108.6 pg/mL, 116.4 pg/mL, 156.8 pg/mL, and 154.7 pg/mL on days 3, 7, 14, and 21, respectively, in the sham operation group. The expressions of the BDNF were 33.62 pg/mL, 32.28 pg/mL, 32.28 pg/mL, and 33.03 pg/mL on days 3, 7, 14, and 21, respectively, in the model group. Moreover, those in the meridian massage group were 47.87 pg/mL, 56.70 pg/mL, 75.70 pg/mL, and 87.70 pg/mL on days 3, 7, 14 and 21 (Figure 4(b)). The above results indicated that meridian massage reduced the expression of miR-206 and increased the expression of BDNF after cerebral infarction.

### 3.4. BDNF Acted as a Target Gene of miR-206

Detection by a dual-luciferase reporter system revealed that the ratio of Renilla luciferase/firefly luciferase was reduced in the miR-206 and BDNF-WT-3′UTR co-transfection group, whereas the ratio of Renilla luciferase/firefly luciferase exhibited a remarkable change in the BDNF-MUT-3′UTR group indicating BDNF served as a target gene of miR-206 (Figure 5(a)). To further verify the effect of miR-206 on the BDNF, we overexpressed or silenced miR-206 in C2C12 myoblast cells (Figure 5(b)). Results of qPCR showed that miR-206 was downregulated in traction tension-treated C2C12 myoblast cells (Figure 5(c)). Overexpression of miR-206 significantly reduced the mRNA level of BDNF, and its level was restored after traction tension treatment, contrary to miR-206 inhibition (Figures 5(d) and 5(e)). Immunofluorescence and western blot at the protein level showed the same expression trend as mRNA (Figures 6(a)–6(d)).

## 4. Discussion

Meridian massage functions as a benign physical stimulus based on scientific research. An external force is provided by massage manipulations working at specific parts and acupuncture acupoints on the body surface. The massage technique is employed to stimulate the body and adjust the functions of corresponding organs [22, 23]. Hemiplegic limb movements are difficult to coordinate mostly due to a unified balance that cannot be achieved in antagonistic activities of the nervous system between excitement and inhibition after cerebral infarction. The abnormal antagonistic functions can be improved through massage manipulations, thereby coordinating the movement of the body extremities. Timely meridian massage and limb function training can speed up motor function reconstruction in the affected limbs, reduce sequelae occurrence, and shorten hospital stay for patients with cerebral infarction. Acupoint massage for these patients with cerebral infarction and hemiplegia can promote the recovery of the affected limbs and facilitate their living ability for the rest of their lives. Rehabilitation training after cerebral ischemia promotes nerve regeneration and the recovery of motor function. The recovery of brain functions can be achieved for a large number of patients because of plasticity changes after brain injury, which presents a theoretical basis for rehabilitation treatment of cerebral infarction [24, 25]. Muscles and joints are moved by rehabilitation training, through which many sensation impulses on the body and skin were input into the central nervous system, stimulating cerebral blood circulation, enhancing excitability of nerve cells in the semidark region around lesions, facilitating recovery and compensation of neuron functions and maximizing the function of reconstruction, thereby promoting the formation of normal functional patterns [26, 27]. By manipulating meridian massage in rats after cerebral infarction, we found in this study that meridian massage effectively improved the morphology and structure of brain tissues and reduced autophagy and apoptosis of brain tissue cells in rats after cerebral infarction, through which an obvious improvement was achieved offering an insight of research guidance for meridian massage application in clinical rehabilitation physiotherapy.

This study testified target relationship and differential expressions between miR-206 and BDNF in the cerebral infarction model group and the meridian massage group by qPCR and WB. As a neurotrophic factor, the BDNF exerts essential roles in the in vivo development of motor neurons, the survival of adult motor neurons, survival of pathological motor neurons, and even the regeneration of axons and protection of brain tissues after ischemia. The BDNF serves notably as the most effective bioactive substance to maintain and protect the survival and growth of motor neurons and is the only one continuously expressed in the central nervous system and peripheral nerve tissues. Furthermore, the successive expression of the BDNF in gastrocnemius muscles after birth indicates a long-term role in promoting the development and maintenance of NMJ function [28, 29]. It is assumed the role in refining the synapse since one was given to birth, which is of great significance for the survival and vitality of nerves. Previous experiments have revealed that appropriate exercise increases the expression of BDNF-promoted functional changes in synapses and assisted the NMJ synaptic function in NTs through presynaptic depolarization [18, 19]. Meridian massage is identical to an exercise that produces constant stimulation on affected areas and induced BDNF expression.

The expression of miR-206 is significantly upregulated with the prolongation of denervation time, whose precursor molecules are associated with the formation of the terminal motor synapses. Hence, miR-206 molecules may be involved in the pathophysiological process of skeletal muscle atrophy [30, 31]. After denervation of skeletal muscle atrophy, some expression changes occur in such muscle-specific miRNAs, miR-206 in particular exhibits a dramatically upregulated expression, thus we speculate that these skeletal muscle-specific miRNAs might act as regulators in the process of denervated skeletal muscle atrophy. A load experiment of skeletal muscle hypertrophy in rats revealed that no change was noticed in the expression of mature miR-206 despite the level of the original miR-206 transcript being highly upregulated. Among rats with muscular dystrophy, the expression of miR-206 in septum presented 4.5 folds higher than that of normal rats, while no change of miR-206 was observed in other skeletal muscles [32]. A high level of miR-206 was seen in newly formed muscle fibers indicating that it may be associated with myogenesis and maturation processes of muscle atrophy.

## 5. Conclusions

This study demonstrates that meridian massage assists in reducing nerve damage and repairing brain tissues to inhibit the expression of miR-206, thereby enhancing the expression of the BDNF. Our findings further reveal that the restoration of brain structures and functions after cerebral infarction can be promoted through successive meridian massage, which is expected to provide a certain research insight for TCM application in cerebral infarction recovery and treatment. It provides a theoretical basis for the clinical application of meridian massage, but the mechanism of action is not yet fully understood, which will be the goal of further research.

## Figures and Tables

**Figure 1:** Cerebral infarction model in rats and HE staining. (a) Schematic diagram of cerebral infarction model operation; (b) cerebral infarction area; (c) HE staining to detect the hippocampus area and cortical area.

**Figure 2:** Transmission electron microscopy detection of rat nerve cells. Yellow arrows represent apoptotic cells; red arrows represent swollen mitochondria; green arrows represent intracytoplasmic vacuole; blue arrows represent autophagy.

**Figure 3:** qPCR detection of the miR-206 and BDNF expression in gastrocnemius muscle and whole blood. (a) miR-206 expression in whole blood; (b) BDNF expression in whole blood; (c) miR-206 expression in gastrocnemius muscle; (d) BDNF expression in gastrocnemius muscle.

**Figure 4:** The Western blot and ELISA results of the BDNF expression in gastrocnemius muscle. a: WB detection; j: Sham; m: cerebral infarction. (a) Treatment group; (b) ELISA detection of BDNF in gastrocnemius muscles; (c) Western blot statistical results.

**Figure 5:** miR-206 acts on the BDNF and downregulates its expression at the mRNA level. (a) Dual-luciferase reporter system to detect the targeting relationship between miR-206 and BDNF. (b) The expression of miR-206 in traction tension-treated C2C12 cells was detected by qPCR. (c, d) Regulation of BDNF expression in C2C12 cells by overexpression or silencing of miR-206. ^##^*P* < 0.01 between two compared groups.

**Figure 6:** miR-206 downregulated BDNF at the protein level. (a, b) BDNF protein level in C2C12 cells was detected by western blot. Relative protein expression was measured by Image J. (c, d) The expression of BDNF was detected by immunofluorescence in C2C12 cells.

## Data Availability

The data used to support the findings of this study are included within the article.
